# Face Detection Algorithm Based on Double-Channel CNN with Occlusion Perceptron

**DOI:** 10.1155/2022/3705581

**Published:** 2022-01-28

**Authors:** Yueying Li

**Affiliations:** College of Information Engineering, Xinyang Agriculture and Forestry University, Xinyang 464000, China

## Abstract

Aiming at the problem of low accuracy of face detection under complex occlusion conditions, a double-channel occlusion perceptron neural network model was proposed. The area occlusion judgment unit is designed and integrated into the VGG16 network to form an occlusion perceptron neural network. Thereupon, the features of unoccluded regions and less occluded regions in facial images are extracted by the perceptual neural network. Transfer learning algorithm is utilized to pretrain parameters of the convolution layer to reduce the overfitting problem caused by insufficient training data samples. Face features of the whole face were extracted by optimizing the residual network, and then the face features of the occluding perceptron neural network and the residual network were weighted and fused. Experiments were carried out on two open data sets, AR and MAFA. The results demonstrate that the detection accuracy of this method is higher than that of other methods, and the detection speed is faster.

## 1. Introduction

As a research hotspot in the field of computer vision, face detection is the basis of face analysis tasks such as face retrieval [1], face alignment [2], human-computer interaction [3], and face superresolution reconstruction [4]. In recent years, Convolutional Neural Network (CNN) [5–7] has made great achievements in the field of unconstrained face detection. Many scholars at home and abroad have also proposed many excellent network structures [8, 9] and loss functions [10, 11]. For example, literature [12] proposes an orthogonal embedded CNN network, which enhances feature learning of age-invariant deep face. Literature [13] put forward a large margin cosine loss function, which improves the discriminant ability of the traditional CNN network softmax layer. The above methods further improve the performance of CNN face detection, some of which even surpass human recognition ability in some specific data sets.

Although the face detection method based on CNN has achieved great success, the depth feature does not have feature invariance under the influence of light, posture, expression, occlusion, and other factors. It is difficult to obtain satisfactory results for face detection under complex occlusion conditions. In real scenes, face images usually have various types of facial occlusion, including sunglasses, masks, scarves, and water glasses, and face features are damaged to a large extent under the influence of occlusion factors. With the improvement of occlusion degree, the difficulty of face detection increases, making it difficult for more advanced face detection methods [14, 15] to accurately determine the location of occluded faces.

Before the emergence of deep CNN, face detection methods under partial occlusion are mainly divided into two categories. The first type of method usually divides the face image into several local regions. During feature extraction, local feature descriptors are only extracted from nonoccluded regions [16, 17]. However, these methods are limited by the performance of shallow features, and the detection performance is weak. The second type of approach focuses on restoring facial features in occluded areas. The most representative method is Sparse Representation Classification (SRC) [18], which uses a linear combination of training images and sparse constraint of occlusion to recover unoccluded faces. Although it improves the detection accuracy, this method is not scalable enough. Besides, it requires high consistency between test data and training data.

In recent years, deep CNN has played a dominant role in occlusion face detection. Literature [19] adopts an active learning strategy to synthesize occlusion face to expand training data, and its detection performance is high. However, this method cannot solve the problem of face detection in essence because the extended training data can only ensure a more balanced extraction of local features. In literature [20], long short-term memory (LSTM) autoencoder was used to restore the blocked area of the face, and the recovered face image was detected. This method can reduce the influence of occlusion to some extent, but it is difficult to ensure the matching of the attributes of the restored area and the unoccluded area in the open scene. In reference [16], MaskNet branches were added to the middle layer of CNN to assign a lower weight to the occlusion area during feature activation, thus reducing the interference of occlusion to detection. However, the MaskNet branch lacks additional oversight information, resulting in insufficient differentiation of the intermediate transformation layer. In conclusion, the shallow feature-based occlusion face detection method has limited recognition ability. However, the method based on deep learning ignores the inconsistencies of two faces under different occlusion conditions and fails to fully consider the influence of occlusion.

The innovations and contributions of this paper are listed as follows:

1. The occlusion problem in face detection is analyzed, and a neural network with occlusion perceptron ability is proposed, which can extract face features in face occlusion.
2. A regional occlusion judgment unit is designed and integrated into the visual geometry group network (VGGNet) [21]. It enables the whole model to extract face features from unexcluded regions and less occluded regions.
3. The parameters of the convolution layer are pretrained by a transfer learning algorithm. Facial features were extracted using the modified residual network based on the residual neural network. Finally, the weighted fusion residual network and the output of the occlusion perceptron network are used for face detection.

The structure of this paper is listed as follows. The related work is described in the next section, which contains the convolutional neural network and feature extraction method. The proposed method is expressed in Section 3. Section 4 focuses on the experiment and analysis. Section 5 is the conclusion.

## 2. Related Work

### 2.1. Network Structure

Convolutional Neural Network (CNN) has made remarkable achievements in the field of computer vision. The main reason for the remarkable achievements in image classification, target detection, and other fields is the continuous improvement of network architecture [22]. For example, Alex Net proposed achieved excellent performance in ImageNet competition (the error rates of top1 and top5 were 37.5% and 17.0%, respectively) [23]. The emergence of Alex Net causes people to study CNN upsurge. Literature [24] designed convolutional neural network to conduct a visual analysis of network interior and further improve CNN capability. Deconvolution neural network is mainly composed of three parts: antipooling, antiactivation, and deconvolution. By visualizing each feature layer of Alex Net, the convolution kernel size and step size are optimized. Compared with Alex Net, the classification error of the improved model in ImageNet 2012 is reduced. VGGNet is proposed, which successfully constructed a 16/19-layer deep neural network by exploring and analyzing the relationship between depth and performance of convolutional neural network [21]. Literature [8] proposed residual convolutional neural network to solve the performance degradation problem when the number of network layers reached a certain level. By adding jump structure to the network to realize identity mapping, it realizes the purpose of using network depth to improve accuracy.

This paper proposes a model architecture based on VGGNet and residual network. The main reason for choosing VGGNet in this paper is its excellent performance in image feature extraction, and it is easy to modify and train. Residual network is used because it is easy to optimize and can extract face features well with a simple modification.

### 2.2. Feature Extraction

Face recognition in the real world is a challenging task in that there are many inevitable problems in the recognition process, such as partial occlusion, illumination variation, individual differences, and so on. All these problems are related to face nonlinearly in spatial expression. Therefore, it is very difficult to extract facial features effectively. In order to solve the various problems encountered in face recognition, researchers try to continuously optimize the network architecture and propose new algorithms to solve them. For example, literature [25] proposed Weighted Mixed Deep Neural Network (WMDNN) model to effectively improve the robustness of the model to light changes. This model can effectively fuse the features of facial gray image and LBP image and successfully construct the light insensitive model. The model proposed in this paper is like this model and adopts dual-channel output fusion to obtain better performance. To solve the problem of occlusion, Krizhevsky et al. [23] proposed Convolution Neural Network with Attention (ACNN) mechanism, which is composed of patch based ACNN (pACNN) and Global based ACNN (gACNN). By perceptron the proportion of occluded areas on the face, the network is focused on unoccluded areas. Different from ACNN, the proposed model uses multiple regional occlusion judgment units to form an occlusion perceptron network, which is easier to train and optimize than ACNN. In order to solve the shortage of sample data, literature [26] proposed the transfer learning algorithm to conduct parameter pretraining for the convolution layer of the face recognition network. The algorithm is a two-stage training algorithm. In the first stage, face information is used as the supervised value of convolutional layer parameter training to realize the initialization of convolutional layer parameters. In the second stage, face information is used as the monitoring value to train the parameters of the full connection layer, to solve the overfitting problem caused by insufficient training data.

The proposed model is mainly aimed at partial occlusion in face recognition. Based on ACNN, the area occlusion decision unit is designed and integrated into a single network. This design enables the network to have an occlusion perceptron function. Dual-channel network structure is adopted to realize feature complementation to obtain better performance. In addition, the transfer learning algorithm is applied to pretrain the network to solve the overfitting problem caused by insufficient training samples.

## 3. The Proposed Method in This Paper

### 3.1. The System Framework

The overall framework of the model proposed in this paper is shown in Figure 1. The occlusion perceptron network is used to extract facial features in fewer occlusion regions. The main function of the Region Decision Unit (RD-Unit) is to determine whether the occlusion ratio of the subregion exceeds the set value. When the occlusion of a certain area exceeds the set proportion, the feature vector of the area is discarded. In this paper, several regional occlusion judgment units are integrated into the VGG16 network to screen out the subregions with less occlusion. Therefore, the occlusion perceptron network can extract the face related features in fewer occlusion areas. Residual neural network (RNN) is applied to extract full-face features. The output of the two networks is fused with feature vectors by the single-factor weighting method, and the fused feature vectors will be used for face detection.

### 3.2. The Occlusion Perceptron Network

In this paper, Face++ is employed to call the application programming interface (API) to detect key points on the face, and the API can be obtained at https://www.faceplusplus.com.cn/face-detection. Then, OpenCV is put used to select the area containing key points in the image (). The face image after processing will be uniformly scaled to 128 pixels × 128 pixels. Then, its services as the input of the occlusion perceptron network for feature extraction. In the feature extraction stage, the sliding partition method is used to select the subregions. Use a fixed size window and set the sliding step, and then use the progressive sliding mode for face image sliding selection.

Assume that the width and height of the input image are W and H, respectively, and the sliding window size is *d* × *d*. After the input image is divided by the sliding partition method, *t* subregions will be obtained. Its calculation equation is as follows:

(1) $$\begin{array}{c} t=\left[\frac{m-d}{s}+1\right]\times \left[\frac{b-d}{s}+1\right], \end{array}$$

where *s* is the size of the sliding step. The experimental results show that the sliding step is proportional to the network accuracy and memory consumption. Overall consideration, this paper sets the sliding step as 1/2 of the sliding window size, that is, *s* = *d*/2. Swiping results in some area overlap and resource consumption, but it helps preserve more of the face. The sliding selection method operates on the whole image and has low dependence on the positioning accuracy of facial key points. Therefore, this method can improve the performance of the occlusion perceptron network to a certain extent. When the size of *d* is set to 32, 49 subregions will be obtained after sliding division on the face image with a size of 128 × 128 pixels. In practice, this classification method is carried out at the level of the image feature graph, and network parameters are reduced by sharing a convolutional layer. The segmented region feature map will be used to extract the face features of the region with less occlusion than the set proportion through the occlusion judgment unit.

The structure of the occlusion perceptron network is displayed in Figure 2. The main function of the network convolution layer is to transform input into a feature graph. It consists of 12 convolution layers and 4 pooling layers. The size of the convolutional layer filter is 3 × 3, and the size of the pooled layer filter is 2 × 2. The main function of the area occlusion judgment unit is to judge the occlusion of the divided area, that is, to judge whether the occlusion proportion of the area exceeds the set proportion threshold. The occlusion judgment unit is composed of two branches. The first branch is the decision network, and the second branch is the full connection layer. The decision network consists of one pooling layer, two full connection layers, and one logistic regression function. The input of the decision network is the regional feature graph, and a one-dimensional vector is obtained after pooling operation and vector feature extraction. Finally, a logistic regression function is used to realize the occlusion judgment of the vectors in this region. If the occlusion ratio of this region exceeds the set threshold, the label of this region is judged to be 0, and the feature vector extracted from the second branch of this region is discarded. If the shielding ratio is less than the set threshold, the feature vector of the region is retained.

In this paper, *ρ*_*x*_ is used to represent the feature map of the ith region. The first branch is the decision network, which can perform occlusion ratio judgment for *ρ*_*x*_.

(2) $$\begin{array}{c} \eta_{x}=\delta \left(\rho_{x}\right), \end{array}$$

where *ρ*_*x*_ represents the judgment result of the *x*-th region. *δ*(·) is a classification function and represents the decision operation in the decision network, as shown in the following equation:

(3) $$\begin{array}{c} \delta \left(i\right)=\left\{\begin{array}{c} 1,\text{Oh}\leq \beta ,\\ 0,\text{other,} \end{array}\right. \end{array}$$

where Oh is the regional occlusion ratio. *β* is to set the threshold of occlusion ratio. 1 indicates that the occlusion ratio in this area is lower than the set threshold. 0 means that the occlusion ratio of this region is judged to exceed the set threshold, indicating that the feature vectors learned from this region will not be fused. Finally, a decision operation is performed on the output of channel *x*.

(4) $$\begin{array}{c} q_{x}=\eta_{x}\times \tilde{\rho_{x}}, \end{array}$$

_where_*ρ*_*x*_ represents the vector representation learned in the second branch full connection layer. *q*_*x*_ represents the regional feature vector after the decision operation.

After experimental analysis, the following results are obtained. When the occlusion ratio was more than 0.5, the accuracy decreased significantly. When the occlusion ratio was less than 0.5, the accuracy also decreased significantly. Therefore, the threshold of occlusion ratio is manually set to 0.5. That is, the feature vectors of regions with occlusion ratio less than 1/2 are reserved for face detection. The feature vectors of the areas with less occlusion will be retained by the occlusion perceptron network through the screening of the occlusion judgment unit.

In this paper, multiple occlusion decision units are integrated into a single neural network, and the region is divided by window sliding. Through the combination of the two methods, the neural network can screen out the areas with less occlusion ratio, thus forming the occlusion perceptron neural network. In addition, the convolutional layer sharing is realized by subregion division in the feature graph to reduce network parameters, to achieve the optimization effect of the model. The parameters of the convolutional layer of the occlusion perceptron network will be pretrained by the transfer learning algorithm FaceNet2ExpNet [26].

### 3.3. The Residual Network

Large area occlusion and nonocclusion can cause the loss of some details in the occlusion perceptron network. Therefore, another deep neural network is exploited to extract full-face features to achieve the complementary effect of masking and perceptron network. The network is based on the residual network which is easier to optimize. The advantage of a residual network is that when the network depth reaches a certain degree, it can be further optimized to improve performance. Unlike ordinary networks, performance degradation will not occur with the increase of network depth because the residual network introduces identity mapping in the two convolution layers. Identity mapping is equivalent to adding short-cut connections in the middle of the network layer to form high-speed branches to form basic residual units. Suppose that the output to be learned is *H(x)* in a residual network *F(x)*. That is, *H(x)−x* will be learned. This means that instead of learning the output *H(x)* of the network, you learn the difference between the output *H(x)* and the input *x*. If the difference value is close to 0, it will indicate that gradient disappearance occurs in this layer network. This means that no valid information is learned in this layer of the network and that the network will be jumped. The network achieves further optimization without introducing additional parameters and increasing computation by means of identity mapping. Residual learning unit applied to the deep convolutional neural network can effectively alleviate the problem of gradient disappearance in network model training, which solves the problems of hard training and performance degradation of the deep network.

In this paper, the residual network is used as the backbone of the second network. The 101-layer residual network was modified to extract the relevant features of full-face images, and the modified network structure was 102 layers. For the first layer of the network, change the size of the 7 × 7 filter to 5 × 5. Because the 7 × 7 filter is relatively large for facial features, it cannot capture details. Subsequently, the filter size of the pooling layer was adjusted accordingly, from 3 × 3 to 2 × 2. The other four convolution blocks still use filters of size 1 × 1 and 3 × 3. Correction Linear Unit (ReLU) is used as the activation function during the convolutional layer training phase, and Batch Normalization (BN) is used to process the activation values. Finally, the 1000-dimensional single full connection layer is changed to two full connection layers, 256 and 64 dimensions, respectively. 256-dimensional vector is put forth to reduce the feature dimension in that 1000-dimensional vector is easy to lead to the overfitting phenomenon for face features. Dropout is applied to further prevent overfitting. Finally, the 64-dimensional vector of the residual network is fused with the output of the occluded perceptron network.

### 3.4. The Pretraining of Convolutional Layer

The transfer learning method is employed to pretrain the network to solve the overfitting problem caused by insufficient training samples. In the training phase of the convolutional layer of the main channel, the transfer learning algorithm FaceNet2ExpNet is used to pretrain the parameters of the convolutional layer. The training process is shown in Figure 3. The training process is divided into two stages. In the first stage, the deep face feature information in the face network is used as the supervision value, which makes learning facial expressions easy. The training loss function Loss of convolution layer is defined as follows:

(5) $$\begin{array}{c} \text{Loss}=\underset{\theta }{\min}a_{\theta }\left(X\right)-A{\left(X\right)}_{u}^{u}, \end{array}$$

where *A*(*X*) represents the convolution layer output of the face network. *a*_*θ*_(*X*) represents the convolution layer output of the face expression network. ‖·‖_u_^*u*^ said regularized training by using *p* paradigm. L2 normal form is used in this paper, and ReLU is used as the activation function in each convolution layer.

In the second stage of training, the parameters of the convolution layer are frozen first. Then, the output of pool5 is used for supervised learning of facial expression network learning. Finally, the full connection layer is added after the convolution layer for training.

### 3.5. The Feature Fusion

After feature extraction of the double network channels is completed, weighted fusion will be performed on the outputs. Single-factor weighting method is adopted in this paper, and its fusion method is shown in Figure 4. The output of the occlusion perceptron network will be equally fused. That is, the effective output of the occlusion judgment unit will be equally weighted fused to obtain a 64-dimensional feature vector. Then, the feature vector is fused with the residual network feature vector by single-factor weighting.

Use *q*_*f*_ to represent a single output of a zone decision unit. *q*_*f*_−_1_ represents the vector obtained after the fusion of all effective feature vectors in the occlusion perceptron network. The eigenvectors are obtained from the fusion of all the vectors whose shielding is less than the threshold subregion transformation. *q*_*f*_−_2_ represents the residual network output vector, and finally, the fusion vector *q*_*f*_ is obtained by single-factor weighted fusion.

(6) $$\begin{array}{c} q_{f}=\alpha \cdot q_{f_{-}1}+\left(1-\alpha \right)\cdot q_{f_{-}2}, \end{array}$$

where *α* is the weighting factor, representing the proportion of the shielding perceptron network output in the fusion vector. The value of *α* ranges from 0 to 1. We classify expressions using the softmax classification function and calculate the probability value ${\hat{j}}_{x}$ for each expression.

(7) $$\begin{array}{c} {\hat{j}}_{x}=\frac{e^{i_{x}}}{\sum_{y=1}^{Z}e^{i_{y}}}Z, \end{array}$$

where *Z* represents the type of face detection. *i*_*x*_ represents the output value of the *x*-th face detection. When training the full connection layer, the cross-entropy loss function will be used to optimize the whole network, and its equation is defined as follows:

(8) $$\begin{array}{c} L\left(j,\right)=\sum_{x=1}^{Z}j_{x}{\text{loa}}_{g}{\hat{j}}_{x}, \end{array}$$

where *j*_*x*_ is the truth tag of face detection and ${\hat{j}}_{x}$ is the prediction tag for face detection.

## 4. Experiment and Analysis

### 4.1. Experimental Configuration

All the experimental data in this paper were obtained on NVIDIA CUDA Framework 6.5, and NVIDIA GTX 1080 GPU was used for the experiment. In addition, VGGNet is used as the backbone network of ACNNs. Image data from the WIDER FACE dataset [27] were used to initialize network parameters. To verify the accuracy and effectiveness of the proposed method, AR face dataset [28] and MAFA occluded face dataset [29] were selected for experiments.

Small batch stochastic gradient descent was used to optimize the model. The basic learning rate was set to 0.001 initially and reduced to 0.1 by a polynomial strategy. Momentum is set to 0.9 and weight attenuation is set to 0.0005. During the training phase, the value of the actual batch size is set to 64 and iterated 10,000 times. When training the residual network, the convolutional layer is pretrained using a FACE image on WIDER FACE and the parameters of all the convolutional layers are initialized. Then, the convolutional layer parameters are fixed and the final fully connected layer is fine-tuned. During the training, the value of the learning rate is set to 0.01. After 20000 iterations, the value of the learning rate was adjusted to 0.0001 in the fine-tuning stage, and another 10000 iterations were carried out. The training of the whole model took 3 days, and it took 1.2 s for the model to process a single image after the parameters were fixed.

### 4.2. Weight Evaluation

In this paper, the weight factor *α* is evaluated on two reference databases. During the test, the initial value of *α* was set to 0 and the increment was set to 0.1. When *α* = 0, it means that only the output of the occluded perceptron network is used as the classification result. When *α* = 1, it means that only the output of the residual network is used as the classification result. As shown in Figure 5, Figures 5(a) and 5(b) represent the evaluation results on the two databases of AR face dataset and MAFA occluded face dataset, respectively. On these two databases, the model achieves the best performance when *α* is 0.7 and 0.6, respectively. Then, the value of *α* was further tested, and the results showed that when *α* was 0.65, the overall performance of the model on the two databases was the best. Therefore, this paper finally sets the value of *α* as 0.65 manually. Figure 5 proves that the output fusion of the two networks can effectively improve the performance of the model.

### 4.3. Experimental Results and Analysis

#### 4.3.1. AR Data Set

The AR face dataset contains more than 4000 color images with different facial expressions, lighting conditions, and face occlusion. They were collected from 126 subjects, including 70 men and 56 women. These images came from two meetings 14 days apart. There were no restrictions on subjects' clothing, makeup, and hair at the time of collection, and the same images were taken for each subject in both sessions. In this paper, images shielded by sunglasses and scarves are selected as test images in the AR face dataset. The experimental results are shown in Table 1.

As can be seen from Table 1, the method presented in this paper improves the accuracy of face detection under the occlusion of sunglasses and scarves while maintaining low time loss. Compared with the other four methods, the detection accuracy of the proposed method is higher, indicating that the detection accuracy of the occluded face can be improved effectively by shielding the face feature element damage caused by local occlusion.

#### 4.3.2. MAFA Data Set

The MAFA Occluded face dataset tagged 35,806 occluded faces in 30,811 images. Each marked face contains six attributes, which are face position, eye position, occlusion position, face direction, occlusion level, and occlusion type. The training set contained 29,452 occluded faces, and the test set contained 6354 occluded faces. The average accuracy pairs of each method on the MAFA test set are shown in Table 2.

In Table 2, various types of face occlusion tests are conducted in this paper. The first test involves multiple face deflection angles. When the face is facing straight forward, the average accuracy of all detection methods reaches their maximum value. However, with the increase of face deflection Angle, the detection difficulty continues to improve, and the average accuracy of all methods decreased significantly. The second type of test includes the shielding level from low to high. With the improvement of the shielding degree, the detection accuracy of each face detection method decreases rapidly. The third type of test consists of a variety of mask types, including simple mask, complex mask, human mask, and mixed mask. The more complex the mask is, the lower the accuracy of mask detection will be. As can be seen from Table 2, the average accuracy of the proposed method is higher than that of other comparison methods in the tests of 3 categories and 12 subcategories. In addition, the detection speed of the proposed method is faster than other methods, which shows that the proposed method can achieve higher accuracy and faster occlusion face detection.

## 5. Conclusion

A double-channel network model with occlusion perceptron capability is proposed in this paper. Firstly, the mask perceptron neural network is designed to extract face image features under occlusion. Then, the optimized residual network is used to extract the features of the whole face image. In the model training stage, the transfer learning algorithm is adopted to pretrain the parameters of the convolution layer. Finally, the double-channel network outputs are fused to further improve the overall model performance. Experimental results on AR and MAFA datasets demonstrate that the proposed method has higher detection accuracy than other compared occlusion face detection methods. The next step is to extend the proposed method to 3D occlusion face detection to solve the problem of depth image occlusion face detection. Since the training of the algorithm in this paper takes a long time, it will also be further analyzed in future work.

## Figures and Tables

**Figure 1:** The proposed framework of this paper.

**Figure 2:** Structure of occlusion perceptron network.

**Figure 3:** The transfer learning in the pretraining process.

**Figure 4:** The weighted fusion of double-channel outputs.

**Figure 5:** Evaluation results of weight factors on different databases. (a) The weight evaluation result on the AR Face database. (b) The weight evaluation result on the MAFA dataset.

**Table 1:** The face detection accuracy in AR dataset.

Method	Accuracy (%)		Speed (FPS)
	Sunglasses shade	Scarf shade	
Literature [14]	91.11	97.54	20
Literature [16]	97.25	98.35	17
Literature [30]	97.57	90.73	35
Literature [31]	95.53	98.62	26
Proposed	99.46	99.73	33

**Table 2:** The average accuracy of face detection in MAFA dataset.

Attribute	Literature [14]	Literature [16]	Literature [30]	Literature [31]	Proposed
Left	3.02	11.8	17.4	14.2	19.9
Left-front	28.7	35.3	46.8	39.5	65
Front	66.8	70.4	76.8	72.6	82.2
Right-front	20.7	25.4	32.6	28.9	59.3
Right	2.07	6.78	17.5	9.94	19.3
Weak	59.6	64	74.9	67.9	80.6
Medium	44.4	49.6	65.7	62.3	72.6
Heavy	7.23	20.8	26.3	22.9	35.8
Simple	64.6	69.7	74.4	71.5	81.6
Complex	51.2	54.7	62.3	57.6	74.9
Body	25.5	30.3	43.2	39.6	65.4
Hybrid	10.8	16.2	21.8	18.5	28.7
Accuracy	62.9	67.4	73.5	69.7	80.2
Speed (FPS)	22	20	38	28	39

## Data Availability

The labeled dataset used to support the findings of this study is available from the corresponding author upon request.
